The article "Evaluating sports complex sustainable supply chains: A prospective assessment technique method of moments quantile regression research" was retracted in 2025. Reasons: concerns about the peer review; concerns about the authorship; concerns about the article.

# Evaluating sports complex sustainable supply chains: A prospective assessment technique method of moments quantile regression research

**DOI:** 10.1371/journal.pone.0323054

**Published:** 2025-06-03

**Authors:** Jialong Liu, Xin Su, Yang Wang

**Affiliations:** 1 Department of Physical Education, Changchun University of Technology, Changchun, Jilin, China; 2 School of Education, Sehan University, Mokpo, Korea; 3 Department of Physical Education, Changchun University of Chinese Medicine, Changchun, Jilin, China; 4 School of Economics and Management, Shanghai University of Sports, Shanghai, China; Nanjing University of Aeronautics and Astronautics, CHINA

## Abstract

The growing emphasis on sustainability in supply chain management has raised critical concerns about its implementation in complex ecosystems such as sports stadiums. This study investigates the economic and environmental dimensions of sustainable supply chains within sports complexes, employing the Method of Moments Quantile Regression (MMQR) technique to provide a nuanced analysis of key variables influencing sustainability outcomes from 2008 to 2022. By integrating Corporate Environmentalism (CE), Population Density (PD), Economic Complexity Ratio, and Workforce Readiness Ratio with Gross Domestic Product (GDP) differentiation metrics, the research identifies significant conditional and non-linear relationships. Results reveal that CE plays a pivotal role in driving GDP differentiation, particularly in lower quantiles, highlighting the potential of sustainability to contribute to balanced economic growth. Population Density consistently influences sustainability outcomes, underscoring the critical role of demographic factors. Additionally, the study exhibit strong macroeconomic and social implications, emphasizing the importance of inclusive strategies for sustainable development. Notably, higher GDP differentiation quantiles reveal trade-offs between economic and environmental goals, presenting challenges for achieving equilibrium. These findings suggest that policymakers and stakeholders should adopt tailored strategies to balance economic and environmental objectives, fostering sustainable practices in sports stadium ecosystems while mitigating disparities across different economic conditions.

## 1. Introduction

Sustainability in supply chain management has become a critical focus for industries worldwide, driven by increasing environmental concerns and the need for resource efficiency [1]. However, applying sustainable supply chain principles in unique and complex ecosystems, such as sports stadiums, presents significant challenges. Sports stadiums are dynamic entities that operate at the intersection of high economic activity, substantial resource consumption, and diverse social interactions [2]. These venues often cater to large crowds and require considerable energy, water, and other resources, leading to substantial environmental footprints [3]. Despite the growing recognition of the need for sustainable practices, there is limited understanding of how such measures impact the broader economic and environmental objectives of these ecosystems [4]. Furthermore, the interplay between corporate environmentalism, demographic factors, economic complexity, and workforce readiness in shaping the sustainability outcomes of sports stadiums remains underexplored [5]. Existing literature often fails to capture the conditional and non-linear relationships between these variables, particularly in the context of GDP differentiation—a crucial indicator of economic balance [6]. This knowledge gap leaves policymakers and stakeholders without adequate frameworks to assess or implement sustainable supply chain strategies that align economic growth with environmental stewardship in sports complexes [7]. The absence of a comprehensive analysis addressing these challenges creates an urgent need for evidence-based approaches to evaluate and optimize sustainable practices in this critical sector [8].

The ecologically and economically sound supply chain processes are imperative in response to China’s extensive industrial sector, characterized by a prolific manufacturing landscape and growing consumer expectations. Sports stadiums are essential to China’s cultural and economic structure [8]. Given thesignificant economic and environmental implications, adopting sustainable supply chains in large-scale enterprises has distinctive problems and possibilities [9]. Therefore, it is imperative to conduct a comprehensive investigation into sustainable supply chain methods in the specific context of sports stadiums in China. Such practices’ economic and environmental benefits make a valuable contribution to the global discussion on sustainability in supply chain management [10]. The logistics include carefully managing the purchase, storage, transportation, and distribution of products and services [11]. The effective management of logistics plays a crucial role in determining the economic resilience and environmental sustainability of the organizations involved [12].

The growing worldwide focus on environmental consciousness and economic prudence has led to a heightened recognition of the need to evaluate and integrate sustainable practices in supply chain logistics [13]. This study evaluates the inherent economic and environmental benefits derived from adopting sustainable supply chain strategies, specifically in the context of sports stadiums [14]. This study examines the complex relationships between environmental responsibility, economic robustness, and logistical efficacy in sports events by integrating the contingent valuation method and the moments’ quantitative regression method [15]. The transformation of green supply chain management throughout the model represented a significant shift towards environmentally conscious logistical strategies [16]. To explore the complex interplay between green logistics and key economic indicators, revealing the significant effects of carbon emissions on several sectors that contribute to the gross domestic product. This research focuses on sports stadiums, which are crucial institutions for implementing sustainable supply chain strategies due to their significant operational scale and wide-ranging impact [17]. Integrating sustainable solutions into companies’ logistical frameworks is of utmost importance due to the significant economic transactions and environmental effects of their operations. Supply chains reveal a range of financial and ecological advantages [17]. From an economic perspective, the pursuit of sustainability is characterized by optimizing resource allocation and improving operational efficiency [18]. Regarding the environment, sustainability catalyzes the preservation and balance of ecological systems. To effectively traverse the complex dynamics of sustainable supply chains in sports stadiums, this research employs a rigorous analytical framework incorporating the contingent valuation method and the method of moments’ quantum regression method [19]. The techniques above provide a systematic examination of the economic and environmental consequences, as well as the resulting advantages, of integrating sustainability into supply chain operations [20].

This study makes significant contributions to the literature on sustainable supply chain management by providing a novel empirical analysis focused on sports stadium ecosystems, a sector that has received limited attention despite its substantial economic and environmental impact. Utilizing data from 2008 to 2022, this research employs the Method of Moments Quantile Regression (MMQR) technique to examine the conditional and non-linear relationships between Corporate Environmentalism (CE), Population Density (PD), Economic Complexity Ratio (lnECR), Workforce Readiness Ratio (lnWRR), and Gross Domestic Product (GDP) differentiation. By focusing on the sports stadium context in the region of Shanghai, China, the study highlights the unique challenges and dynamics of sustainable supply chain implementation in a densely populated and economically vibrant area. Unlike previous studies that often generalize sustainability practices across industries, this research explicitly addresses the intersection of economic growth and environmental stewardship within sports complexes. The findings reveal how demographic and macroeconomic variables influence sustainability outcomes across different quantiles, offering a granular understanding of trade-offs between economic and environmental objectives. Moreover, the study extends the discourse on sustainability by demonstrating the critical role of GDP differentiation as an indicator of economic balance and by identifying the potential of CE to foster equitable growth in sports stadium ecosystems. This research fills a critical gap in the literature by providing region-specific insights and a methodological framework that can be adapted to other contexts, advancing both theoretical understanding and practical applications of sustainable supply chain management.

## 2. Literature review

The emphasis on developing sustainable practices across various industries highlights the pressing need to tackle global environmental challenges [21]. The imperative shift towards sustainable supply chains holds significant importance within the sports sector, particularly in stadium operations. Supply Chain Sustainability (SCS) encompasses a range of practices about suppliers’ sustainability and the transparency of supply chains. The study conducted on sustainable supply chains holds in terms of bolstering sports stadiums’ ecological and financial aspects [22]. When evaluating the ecological footprint of stadiums, it is crucial to prioritize environmental outcomes, particularly carbon emissions [23].

Moreover, it is imperative to highlight the significant impact of Energy Consumption Reduction (ECR) as an essential outcome. This study highlights the importance of assessing energy consumption in kilowatt-hours (kWh) to evaluate the effectiveness of these sustainable measures [24]. Furthermore, it is imperative to acknowledge that Waste Reduction and Recycling Rates play a pivotal role as fundamental indicators in assessing the overall sustainability of a given system or process [25]. Implementing efficient waste management strategies in sports stadiums mitigates their ecological footprint and yields economic benefits through cost reduction in waste disposal and the exploration of revenue opportunities from recycling [26]. Sports stadiums, as significant infrastructural entities, exert a crucial influence on the formation of societal perceptions and attitudes. Sustainable supply chains within the context of sports stadiums encapsulate a profound legitimate compulsion and effectively deal with a range of pressing environmental and economic difficulties [27,28], including waste management, energy consumption, and the accompanying financial implications. The challenges are multifaceted, influencing various operational aspects of the stadiums and their broader societal significance [29].

The primary emphasis surrounding stadiums has predominantly revolved around entertainment and financial viability. In recent years, there has been a notable transition towards sustainability [30]. Stadiums are increasingly establishing new standards by implementing a range of sustainable practices, such as integrating energy-efficient lighting systems, implementing comprehensive waste reduction programs, and adopting renewable energy sources [31]. While it is crucial to prioritize environmental considerations, it is equally important to acknowledge the significant economic implications associated with sustainability. The adoption of sustainable supply chains has the potential to yield substantial financial advantages. These include reducing operational costs and generating increased revenues through sustainable partnerships and branding. Scholars employ various methodological approaches to the economic and environmental benefits of sustainability in stadiums [31]. The Contingent Valuation Method and the Method of Moments Quantile Regression have gained recognition for their robustness in this context. The methodologies mentioned above offer dependable estimations of both quantifiable and non-quantifiable advantages, rendering them particularly pertinent for all-encompassing evaluations in the context of sports arenas [32]. The sustainability matrix is subject to the influence exerted by the specific nature of the sports events hosted by a stadium [33]. In addition, it is essential to consider various factors involving the stadium’s age, infrastructure quality, and geographical location, as these elements significantly influence the formulation and effectiveness of sustainability strategies [34]. The Gross Domestic Product (GDP), which serves as a measure of regional economic vitality, can potentially impact the allocation of resources towards sustainability initiatives [35]. Simultaneously, a review of population density provides valuable insights into the patterns of urbanization, thereby illuminating the dynamics of local resource availability and consumption. Despite significant advancements in sustainable research about sports stadiums, notable gaps exist, specifically in incorporating economic and environmental metrics [36]. The existing body of research has predominantly concentrated on analyzing either one of these dimensions independently, thereby underscoring the necessity for a comprehensive approach [37]. This study efforts to make up this gap by integrating each of them [38].

### 2.1. Theoretical justification

With increased global awareness, sustainability is a practical need. The discussed transition is grounded in the Triple Bottom Line framework, a comprehensive approach emphasizing financial advantages, environmental sustainability and social equality [39]. The framework above exhibits a notable resonance within various domains, including sports stadiums [40]. These immense infrastructures, which attract substantial public interest and require significant resources, function as microcosms of our development [41]. The operational and managerial strategies employed by the organization align with the intricacies and difficulties associated with urban sustainability theories, emphasizing the importance of maintaining a careful equilibrium between consumption and conservation [42].

Nevertheless, it is essential to note that sustainability encompasses more than just being environmentally conscious [43]. Considering the theoretical framework of the Resource-Based View (RBV), it becomes evident that establishing sustainable supply chains within stadiums goes beyond being merely ethical assets; instead, it assumes a role [43]. They possess the potential to serve as drivers of competitive advantage, thereby stimulating the creation of economic value, enhancing brand perception, and developing reliability among participants. The Contingent Valuation Method (CVM) is a widely recognized economic research technique employed to estimate the economic value of non-market goods and services [44]. The economic theories assert that even intangible environmental advantages that lack a direct market representation, such as improved air quality or carbon neutrality, possess an inherent monetary worth as perceived by individuals [45]. The extensive scope and fluctuating results in a dynamic environment such as a stadium require a more intricate methodology. The sustainability initiatives and their subsequent effects are intricately connected to the socio-economic landscape of the region [46,47]. The theories put in the field of regional economics serve as a reminder that variables such as regional GDP and population density play a significant role in not only setting the stage but also actively influencing and providing context to the journey toward sustainability [48] Economic researchers have observed that various factors, such as resource allocation, stakeholder expectations, and the feasibility of sustainability initiatives, can be significantly influenced by certain entities [49].

Despite a growing body of research on sustainable supply chain management, particularly in industries with high environmental and economic impacts, significant gaps remain when it comes to understanding and addressing sustainability in the context of sports stadium ecosystems [50]. First, much of the existing literature on sustainable supply chains focuses on traditional industries such as manufacturing, retail, and logistics, leaving sectors like sports facilities underexplored. Sports stadiums represent a unique blend of economic activity, resource consumption, and social engagement, creating distinct challenges for implementing and assessing sustainable practices [51]. This lack of focused research limits the understanding of how supply chain sustainability principles can be adapted to address the complex, high-demand nature of stadium operations [52,53].

Second, most studies emphasize linear relationships between sustainability drivers and outcomes, often failing to account for the conditional and non-linear interactions that can occur in real-world systems [54–56]. The dynamic interplay between variables such as Corporate Environmentalism (CE), Population Density (PD), Economic Complexity Ratio (lnECR), and Workforce Readiness Ratio (lnWRR) with Gross Domestic Product (GDP) differentiation remains poorly understood. These non-linear effects are critical for understanding the trade-offs and synergies between economic growth and environmental objectives, particularly in quantile-specific contexts, which have not been adequately explored in prior research [57].

Third, while previous studies have highlighted the importance of demographic and macroeconomic factors in shaping sustainable outcomes, they often neglect the integration of such variables in a unified analytical framework [58]. Variables like population density and workforce readiness are frequently examined in isolation rather than in conjunction with economic and environmental factors. This fragmented approach overlooks the systemic nature of supply chain sustainability, particularly in highly interconnected environments like sports stadiums, where economic, social, and environmental dimensions converge [59].

Another significant gap lies in the geographic and temporal focus of prior research. Much of the existing work is concentrated on regions with advanced economies and well-established sustainability policies, offering limited insights into regions like China, where rapid urbanization, high population density, and evolving economic structures present unique sustainability challenges [60]. Additionally, there is limited longitudinal analysis of how sustainability practices evolve over time in response to shifting economic, demographic, and environmental conditions [61]. The absence of such temporal insights restricts the ability to design adaptive, forward-looking strategies for sustainable supply chains [62].

Finally, most studies focus primarily on the economic or environmental dimensions of sustainability, often treating them as separate objectives. There is a lack of comprehensive research examining the trade-offs between these dimensions, particularly in the context of GDP differentiation, which is a critical indicator of economic equity and balance [63]. Understanding these trade-offs is essential for policymakers and stakeholders to develop strategies that simultaneously advance economic and environmental goals in a sector as resource-intensive and socially significant as sports stadiums [64].

Addressing these gaps requires a multidimensional, region-specific, and dynamic approach that integrates diverse factors influencing sustainable supply chains in sports ecosystems [65]. This study aims to fill these gaps by employing advanced analytical methods, such as Method of Moments Quantile Regression (MMQR), to uncover the complex and conditional relationships between sustainability variables, offering insights that can guide policy and practice in this critical but underexplored domain.

## 3. Data and methodology

### 3.1. Econometric estimation

#### 3.1.1. β-convergence model based on OLS.

The -convergence concept (Haseeb et al., 2021), which covers the unqualified and contingent -convergence models, is used in this work to investigate the convergence of food insecurity. The model for conditional-convergence analysis is as follows.


$$\mathrm{\backslash [}\frac{\begin{array}{c} n\\ 0 \end{array}}{\eta }ln(\frac{CEi_{t}}{CEi_{\left(t-\eta \right)}})=\alpha_{i}+\beta_{0}lnSCSi_{\left(t-\eta \right)}+\varepsilon_{it}\mathrm{\backslash ]}$$

When is the duration of both periods? It may be any positive number greater than 0; in this study, it is assumed to be 0 to allow the maximum amount of data to be included in the econometric investigation (Jia et al., 2023). Measurement (0)‘s regression coefficient, which expresses the yearly growth rate of malnutrition in year t, refers to the second-order differences in food poverty after calculating the following equation.


$$\;\Delta lnEP_{it}=ln(ECRi_{t}/WRRi_{\left(t-0\right)})$$ (1)

Then, equation (0) can be converted into an equation.


$$\Delta lnCEi_{t}=\alpha_{i}+\beta_{0}lnECRi_{\left(t-0\right)}+\varepsilon_{it}$$ (2)

When integrand is the aggregate amount and represents the first-order differential, CE stands for “malnutrition for the specific nation I in year t.” I stand for the nation’s response variable. It is a mistaken word. 0 determines whether the annual rate of food insecurity increase corresponds to or separates the given data. It indicates the lagged effect on the yearly rate of increased malnutrition (Koenker & Bassett, 2007). If 0 is negatively significant, there’s no evidence for absolute interconnection, and the increased countries could reduce undernourishment at a discernible rate. At the same time, all other economies will typically have similar poverty rates. On the other hand, if 0 is significant and positive, then there is no substantiation for absolute integration. To investigate the possibility of a conditionally -convergence development for Food insecurity.


$$\Delta lnTSEi_{t}=\alpha_{i}+\beta_{0}lnGDPi_{\left(t-0\right)}+\sum_{j=2}^{p}n\beta_{j}\ln C_{j,it}+\varepsilon_{it}$$ (3)

#### 3.1.2. Convergence model based on quantile regression.

The conventional mean estimates, or OLS, primarily examine the effects of independent variables on the conditional methods of the predictor variable while supposing that parameters are consistent with the standard normalization requirements. Hence, the conventional mean estimation method only considers the dependent sources. List normal distribution; in other words, Serial correlation only emphasizes the project’s average, which only partially reflects the implicit references. List description and ignores the influence of independent variables on the entire distribution (Machado & Santos Silva, 2019). Therefore, outliers might easily have an impact on the OLS estimate findings. The MMQR estimate is used to calculate this same convergence framework to consider the macroeconomic variability of the undernourishment convergence (Afranie et al., 2019). This estimate does not explicitly rely on the hypothesis of a standard deviation and is appropriate for short data periods (Sala-i-Martin, 1996). The MMQR approximation helps identify possible unobserved heterogeneous links between lags in Food insecurity and its increase at the conditional level, in addition to accounting for the influence of outlier occurrences. The ability to capture the macroeconomic variability of the undernourishment convergent at various considerations probabilities of undernourishment is one of the critical benefits of something like the MMQR approximation.


$$\Delta \ln GDP=\alpha_{i}+\beta_{0}lnWRRi_{\left(t-0\right)}+(\delta_{i}+Z_{it}^{\prime }\gamma )U_{it}$$ (4)

$$Q_{\Delta lnEP_{it}}(\tau |lnCEi_{\left(t-0\right)})=(\alpha_{i}+\delta_{i}q(\tau ))+\beta_{0}lnSCSi_{\left(t-0\right)}+Z_{it}^{\prime }\gamma q(\tau )$$ (5)

$$Q_{\Delta lnEP_{it}}\left(lnCEi_{\left(t-0\right)}\right)=\left(\alpha_{i}+\delta_{i}q(\tau )\right)+\left(\beta_{0}+\gamma q(\tau )\right)lnWRRi_{\left(t-0\right)}$$ (6)

minq∑inx∑tnxρτ(R^it−(δ^i+Zit′γ^)q)

R^it=ΔlnCEit−α^i−β^0lnECRi(t−0) (7)

$$\Delta lnPDi_{t}=\alpha_{i}+\beta_{0}lnSCSi_{\left(t-0\right)}+\sum_{j=2}^{p}n\beta_{j}\ln C_{j,it}+(\delta_{i}+Z_{it}^{\prime }\gamma )U_{it}$$ (8)

$$Q_{\Delta lnEP_{it}}(\tau |X_{it})=(\alpha_{i}+\delta_{i}q(\tau ))+\beta_{0}lnGDPi_{\left(t-0\right)}+\sum_{j=2}^{p}n\beta_{j}\ln C_{j,it}+Z_{it}^{\prime }\gamma q(\tau )$$ (9)

The unrestricted --convergence examination on MMQR is identical to the previous variable selection and estimate process (Barro, 1992).

### 3.2. Data sources

In our research into the dynamics of sustainable supply chains within sports stadiums in China from 2008 to 2022, we have developed a framework comprising various distinct and interconnected variables. At the core of our investigation lies the Carbon emission (CE), which refers to the concrete environmental benefits of implementing sustainable supply chains primarily focused on reducing carbon emissions. However, the hypothesis is that these consequences’ extent heavily depends on the Supply Chain Sustainability (SCS) index. The index above is a comprehensive measure of the area where sustainability integration is observed within the stadium’s supply chain, explicitly focusing on Supplier Sustainability Practices (SSP). In addition, it is essential to note that the environmental impact is being closely examined through the implementation of the Energy Consumption Reduction (ECR) and Waste Reduction and Recycling Rates (WRR) metrics. The former metric quantifies the efficiencies of energy conservation, usually measured in millions of kilowatt-hours (kWh). At the same time, the latter provides a percentage representation of the effectiveness of waste management practices within stadiums.

In addition to considering the primary variables, our study recognizes the significant influence of the nature of sports events, represented by the Type of Sports Events Hosted (TSE) variable. Acknowledging that various events, such as football and basketball, can impose varying pressures on the sustainability infrastructure is essential. To situate our findings within the comprehensive socio-economic fabric of the region, we have included two control variables: Gross Domestic Product (GDP) and Population Density (PD). The former, believed to reflect the region’s economic conditions, is hypothesized to impact sustainability investments’ financial viability and potential profitability. Simultaneously, population density (PD), which measures how crowded an area is and how its inhabitants are distributed across space, may have significant implications for how resources are consumed and the pressures on infrastructure. Table 1 shows the list of selected variables.

**Table 1:** Study variables.

Dependent	Variable Symbol	Description	Unit of measurement
Dependent	Environmental Outcome (CE)	Represents the environmental outcomes related to sustainable supply chains in sports stadiums. It could include reductions in carbon emissions, energy consumption, or waste diversion rates.	Carbon Emissions Reduction
Independent	Supply Chain Sustainability (SCS)	Captures the sustainability practices in the stadium’s supply chain, including supplier sustainability practices and supply chain transparency.	Supplier Sustainability Practices (SSP)
Environmental	Energy Consumption Reduction (ECR)	Measures the reduction in energy consumption achieved through sustainability efforts. It could be measured in units of energy (e.g., kWh) and represents the stadium’s energy efficiency.	1000,000 kWh reduction in energy consumption
	Waste Reduction and Recycling Rates (WRR)	Quantifies the effectiveness of waste reduction and recycling programs in the stadium. It is typically expressed as a percentage of waste that is recycled or diverted from landfills.	60% waste diversion rate
Sports	TSE	The type of Sports Events Hosted (TSE) is a categorical variable capturing the sports events regularly hosted at the stadium. Categories could include football, baseball, soccer, basketball, etc.	
Control	GDP(Gross Domestic Product)	Represents the total economic output of the region where the stadium is located. It is typically measured in currency (e.g., USD) and indicates regional economic activity.	$4,000,000 GDP per capita
	Population Density (PD)	Measures the number of people living in the region relative to its land area. It is typically expressed as people per square kilometre or square mile and can provide insights into urbanization and resource usage patterns.	0,000 people per square kilometre

## 4. Results and discussion

### 4.1. Preliminary test on the normal distribution of variables

The Asian member nations have been hindered from emission reduction from very rapidly expanding forms of transport by a lack of aggressive policies. Public transport contributed 26% of the nation’s Emissions of carbon dioxide in 2008, as well as the lowest deployment of alternatives of any economic inter – and intra inAsia. In 2008, it was predicted that by 2040, nitrogen dioxide (no2 (NOx) emissions, which are caused mainly by using oil for transport, will increase by 40%. Table 2 presented the descriptive statistics.

**Table 2:** Descriptive statistics of the variable.

Variable	Observations	Mean	Std. Dev.	Min	Max
CE	960	00.88	4.68	0.08	2.08
SCS	960	20.40	6.04	0.08	4.28
ECR	960	28.28	4.20	0.28	2.28
WRR	960	68.60	2.62	4.60	6.02
TSE	960	28.20	6.60	4.00	8.20
GDP	960	2.080	0.68	0.08	2.60
PD	960	4.048	0.20	2.48	2.00

The results shown in Table 3 show the Shapiro-Francia and Shapiro-Wilk tests. The Environmental Outcome scaled by GDP (CE/GDP) shows a consistent lack of normality in all samples, which significantly affects the reliability of the parametric methods used in the later levels of the model. The Type of Sports Events (lnTSE) variable demonstrates a surprising outcome in the ‘Non-target country’ category, with a Shapiro-Francia p-value of 0.468***. Population Density (PD). Although the PD variable typically deviates from normality, it appears to have a distribution closer to normal in the ‘Target-country’ sub-sample. The affects the model by considering the potential for heteroscedasticity or other distributional variance related to geographical categorization. Energy Consumption Reduction (lnECR) and Waste Reduction and Recycling Rates (lnWRR) show statistically significant p-values, although these values differ among categories. As an economics researcher, it is interesting that the Shapiro-Wilk test value of 0.664*** in the ‘All’ category stands out and is significantly evaluated for its values in other subsets. Table 3 shows the normal distribution findings.

**Table 3:** Test results for the normal distribution of variables.

variables	Shapiro-Francia test			Shapiro-Wilk test		
	All	Target-country	Non-target country	All	Target-countries	Non-target country
(CE/GDP)	0.840^***^	0.820^***^	0.840^***^	0.840^***^	0.820^***^	0.840^***^
lnTSE	0.880^***^	0.870^***^	0.468^***^	0.820^***^	0.880^***^	0.860^***^
PD	0.870^***^	0.858	0.860^***^	0.883^***^	0.886	0.866^***^
lnECR	0.800^***^	0.868^***^	0.864^***^	0.866^***^	0.860^***^	0.840^***^
lnWRR	0.860^***^	0.838^***^	0.844^***^	0.664^***^	0.888^***^	0.820^***^

•Note=

*Indicates statistical significance at the 10% level.

**Indicates statistical significance at the 5% level.

***Indicates statistical significance at the 1% level.

Table 4 demonstrates the complex links between supply chain sustainability, environmental consequences, and sports stadium performance metrics. The ecological outcome (CE) variable significantly impacts economic performance in Step 1 (β = 0.046, p < .05). Early environmental measures, generally integrated into sustainable supply chains, may enhance economic indicators. With coefficients from 0.408 to 0.622, supply chain sustainability (SCS) positively correlates with financial success but is insufficient. This early data reveals an intriguing subject for further research into supply chain sustainability practices and financial success, even if it is not statistically robust. More variables enhance the model’s explanatory ability, as seen by F-values and Adjusted R^2. In the later phases, SCS and CE are less critical, suggesting that various variables may complicate and impact their effects. Environmental performance, CE, and ECR coefficients are insignificant, making their potential implications challenging to assess. In Step 4, a significant interaction term between CE and another variable (β = 0.044, p < .05) suggests a complex and conditional connection. This dependent effect should be studied, specifically how sustainability policies affect environmental performance. The statistical significance of CE is significant in Step 1 (β = 0.066, p < .05) and decreases somewhat in succeeding stages (p < .10), indicating a persistent impact. The link between early environmental effects and sports performance becomes complicated when additional elements are included. While not statistically significant, the negative coefficients of the Type of Sports Events Hosted (TSE) reveal an intriguing association that needs further study. Correspondingly, the quantile regression findings are reported in Table 4.

**Table 4:** Quantile regressions.

Variables	Economic performance				Environmental performance				Sports performance			
	Step 1	Step 2	Step 3	Step 4	Step 1	Step 2	Step 3	Step 4	Step 1	Step 2	Step 3	Step 4
CE	0.046*	0.084	0.060	0.066	0.080	0.022	0.024	0.026	0.066^*^	0.002^+^	0.028^+^	0.046^+^
SCS		0.428	0.408	0.622		0.268 ^***^	0.202 ^***^	0.264 ^***^		0.282 ^***^	0.284^*^ ^**^	0.286 ^***^
ECR			0.046	0.066			−0.022	−0.006			−0.008	−0.020
WRR			0.082	0.068			−0.042	−0.062			0.006	0.000
TSE			−0.026	−0.028			0.042	0.044			−0.066	−0.060
SCS × ECR				0.002				0.026				0.008
GDP				−0.062				−0.082				−0.024
CE×				0.046				0.044^*^				0.060
F for the step	4.066 ^*^	86.064 ^***^	0.266	0.408	0.642	04.286 ^***^	0.660	2.062	4.864 ^*^	28.442 ^***^	0.882	0.868
F for the regression	4.428 ^*^	44.662 ^***^	20.682 ^*^	02.860 ^**^	0.088	20.066 ^***^	4.242 ^***^	4.862 ^***^	4.442 ^*^	08.422 ^*^	8.244 ^***^	4.662 ^***^
Adjusted R^2^	0.044	0.226	0.266	0.422	0.002	0.066	0.204	0.088	0.002	0.008	0.024	0.042

•Note=

*Indicates statistical significance at the 10% level.

**Indicates statistical significance at the 5% level.

***Indicates statistical significance at the 1% level.

Table 5 shows the economic and environmental impact of sustainable supply chains. This research examines these associations’ complex dynamics using unconditional quantile regressions. We may examine economic ramifications using GDP, the dependent variable. The Environmental Outcome variable (CE at t-0) has a consistent negative trend from the 5th to 7th quantiles. The coefficients become statistically significant at the 5th, 6th, and 7th quantiles (β = −0.040, p < .01, β = −0.060, p < .001). As GDP divergence advances, environmental impact worsens. In higher quantiles, economic and environmental goals may conflict. To emphasize supply chain management balance. This considerable variation shows that exogenous causes or unobserved variables may affect GDP differences differently. This research did not address additional variables or policy frameworks. However, they may affect the result variable at various quantiles (Table 5).

**Table 5:** Unconditional analysis of economic and environmental value of sustainable supply chains.

Variables	1st	2^nd^	3^rd^	4^th^	5^th^	6^th^	7^th^
CE(t − 0)	0.040	−0.0002	−0.020	−0.028	−0.040^**^	−0.060^**^	−0.060^***^
						
	−0.040	−0.020	−0.020	−0.008	−0.008	−0.008	−0.020
Constant	−0.240^***^	−0.040^**^	−0.040	0.008	0.068	0.020^***^	0.080^***^
	−0.08	−0.068	−0.048	−0.04	−0.04	−0.04	−0.048
Observations	008	008	008	008	008	008	008

•Note=

*Indicates statistical significance at the 10% level.

**Indicates statistical significance at the 5% level.

***Indicates statistical significance at the 1% level.

Quantile regressions (dependent variable: the differentiation of GDP).

### 4.2. Conditional analysis

Investigating Table 5 shows that the coefficients for Environmental Outcome (CE) display significant variation across various quantiles. Specifically, they range from 0.040 in the first column to −0.060*** in the seventh column. The *** indicates that the variable is highly significant at the 1% level, suggesting an essential negative relationship between CE and the differentiation of GDP. This influence from a positive to a negative coefficient across different levels indicates an intricate and non-linear connection between CE and GDP differentiation. The range from −0.240*** to 0.080*** suggests different baseline economic conditions across the seven models. These constants should not be overlooked as they provide a solid foundation that accounts for other unmeasured factors influencing GDP variation. The Population Density (PD) consistently emerges as a significant variable with negative coefficients in all seven models (Table 6). The variable is particularly substantial, which enhances the robustness of the model by emphasizing the significance of the population density as an influencing variable in evaluating the impact of CE on GDP differentiation.

**Table 6:** Conditional analysis on Quantile regressions.

Factors	1^st^	2^nd^	3^rd^	4^th^	5^th^	6^th^	7^th^
CE(t − 0)	−0.020	−0.080^**^	−0.088^***^	−0.008^***^	−0.040^***^	−0.048^***^	−0.008^***^
	0.068^*^	0.240^***^	0.260^***^	0.288^***^	0.220^***^	0.228^***^	0.248^***^
PD	−0.660^**^	0.628^***^	−0.640^***^	−0.628^***^	−0.620^***^	−0.622^***^	−0.620^***^
	−0.24	0.066	−0.06	−0.048	−0.048	−0.048	−0.060
Constant	−0.004	0.068^**^	−0.088^***^	−0.020^***^	−0.040^***^	−0.068^***^	−0.008^***^
	−0.04	−0.040	−0.028	−0.020	−0.020	−0.020	−0.040
Panel B	0.008^*^	0.240^***^	0.260^***^	0.288^***^	0.228^***^	0.260^***^	0.280^***^
CE(t − 0)	0.020	0.008	−0.002	−0.002	−0.020^*^	−0.008^**^	−0.020^***^
	−0.820^***^	−0.660^***^	−0.628^***^	−0.622^***^	−0.680^***^	−0.660^***^	−0.640^***^
PD	−0.248	−0.008	−0.080	−0.060	−0.048	−0.048	−0.060
	−0.006	−0.068^**^	−0.000^***^	−0.040^***^	−0.060^***^	−0.080^***^	−0.088^***^
lnECR	0.048	0.220^***^	0.260^***^	0.288^***^	0.220^***^	0.260^***^	0.280^***^
	0.008	0.006	−0.002	−0.000	−0.020^*^	−0.008^**^	−0.020^***^
Constant	0.002	−0.028	−0.048	−0.080	−0.000	−0.008	−0.044^*^
	0.822	−0.460	−0.422	−0.222	−0.208	−0.020	−0.002
Panel C	−0.602	−0.48	−0.420	−0.28	−0.28	−0.268	−0.288
CE(t − 0)	960	960	960	960	960	960	960

•Note=

*Indicates statistical significance at the 10% level.

**Indicates statistical significance at the 5% level.

***Indicates statistical significance at the 1% level.

In the investigation of Table 7, the panel regressions investigate the impact of various factors on Gross Domestic Product (GDP), mainly focusing on Corporate Environmentalism (CE) and Population Density (PD). In Panel A, there are varying levels of significance and effect size observed across the seven models. Interestingly, in the third to sixth models, CE becomes significant at the 1% level with negative coefficients, indicating a robust inverse relationship with GDP differentiation. It appears that as Corporate Environmentalism rises, there is a decrease in GDP differentiation. At the same time, the coefficients for PD consistently show a negative and highly significant relationship at the 1% level in all models. To supports the idea that higher population density is associated with a decrease in GDP differentiation. Once again, the study reveals that CE plays a crucial role, showing negative coefficients that further emphasize its detrimental impact on the differentiation of GDP. The ‘lnECR’ variable shows different levels of significance.

**Table 7:** Asymmetric Quantile regression analysis results.

Factors	1^st^	2^nd^	3^rd^	4^th^	5^th^	6^th^	7^th^
Panel A							
CE(t − 0)	−0.020	−0.080^**^	−0.088^***^	−0.008^***^	−0.040^***^	−0.048^***^	−0.008^***^
	0.068^*^	0.240^***^	0.260^***^	0.288^***^	0.220^***^	0.228^***^	0.248^***^
PD	−0.660^***^	−0.628^***^	−0.640^***^	−0.628^***^	−0.620^***^	−0.622^***^	−0.620^***^
	−0.004	−0.068^**^	−0.088^***^	−0.020^***^	−0.040^***^	−0.068^***^	−0.008^***^
Constant	0.008^*^	0.240^***^	0.260^***^	0.288^***^	0.228^***^	0.260^***^	0.280^***^
	0.020	0.008	−0.002	−0.002	−0.020^*^	−0.008^**^	−0.020^***^
Panel B							
CE(t − 0)	−0.820^***^	−0.660^***^	−0.628^***^	−0.622^***^	−0.680^***^	−0.660^***^	−0.640^***^
	−0.006	−0.068^**^	−0.000^***^	−0.040^***^	−0.060^***^	−0.080^***^	−0.088^***^
PD	−0.040	−0.040	−0.028	−0.020	−0.020	−0.020	−0.020
	0.048	0.220^***^	0.260^***^	0.288^***^	0.220^***^	0.260^***^	0.280^***^
lnECR	0.008	0.006	−0.002	−0.000	−0.020*	−0.008**	−0.020^***^
	0.002	−0.028	−0.048	−0.080	−0.000	−0.008	−0.044^*^
Constant	0.822	−0.460	−0.422	−0.222	−0.208	−0.020	−0.002
	960	960	960	960	960	960	960

•Note=

*Indicates statistical significance at the 10% level.

**Indicates statistical significance at the 5% level.

***Indicates statistical significance at the 1% level.

### 4.3. Robustness analysis

Table 8 shows the study of conditional β-convergence. This table analyzes four main Corporate Environmentalism (CE) models, revealing varying coefficient signs and statistical significance. The negative coefficients show effectiveness at 5% and 1%. Companies prioritizing environmentalism may delay conditional β-convergence, resulting in a more thorough analysis. Population Density (PD) coefficients are constantly positive, with statistical significance at 5% and 1% from the third model. These results show that higher population density leads to faster conditional β-convergence, making it essential to consider in policymaking. The log of Economic Complexity Ratio (ECR) is necessary. From the third to the seventh model, the variable’s significance level rises from 10% to 1%. The variable remains negative throughout. A greater degree of economic complexity may hinder conditional β-convergence, supporting the validity of this approach. The Workforce Readiness Ratio (lnWRR) log shows negative coefficients and varied significance (Table 8). From the third model, it becomes statistically significant at 10% and rises to 1% by the seventh. A negative correlation exists between workforce preparation and conditional β-convergence, complicating the interplay of components.

**Table 8:** Conditional β-convergence analysis.

Variable s	1^st^	2^nd^	3^rd^	4^th^	5^th^	6^th^	7^th^
CE(t − 0)	0.048	−0.060	−0.020^**^	−0.066^**^	−0.220^**^	−0.240^**^	−0.288^***^
	0.088	−0.068	−0.048	−0.06	−0.048	−0.048	−0.06
PD	0.060	0.080	0.260^**^	0.202^***^	0.248^***^	0.286^***^	0.440^***^
	0.008	−0.020	−0.022	−0.088	−0.088	−0.088	−0.066
lnECR	−0.022	−0.028	−0.040^*^	−0.040^**^	−0.028^**^	−0.028^***^	−0.040^***^
	−0.020	−0.008	−0.020	−0.020	−0.020	−0.020	−0.020
lnWRR	−0.020	−0.220	−0.248^*^	−0.288^**^	−0.222^**^	−0.260^***^	−0.288^***^
	−0.228	−0.08	−0.060	−0.028	−0.040	−0.028	−0.040
Constant	−0.060	0.208	0.422	0.688	0.640	0.828^*^	0.066^**^
	−0.820	−0.688	−0.488	−0.460	−0.420	−0.420	−0.440
Obs	920	920	920	920	920	920	920

•Note=

*Indicates statistical significance at the 10% level.

**Indicates statistical significance at the 5% level.

***Indicates statistical significance at the 1% level.

### 4.4. Discussion

The study explores sustainable supply chains’ economic and environmental aspects in sports stadiums [66]. One of the key themes in your findings is the trade-off between financial performance and environmental sustainability. In addition, Population Density (PD) consistently appears as a significant mediating factor in your models, indicating that demographic and spatial characteristics greatly influence sustainability practices [67]. In addition, the concept of Corporate Environmentalism (CE) adds another level of intricacy. Based on the available data, there seems to be a connection between sustainable supply chains and economic indicators [68]. However, the relationship between CE and these metrics is not straightforward and depends on various factors. The relationship between Corporate Environmentalism and economic growth is much more complex than initially thought, affecting the rates of conditional β-convergence and, consequently, the speed at which economies come together to reach a typical steady state [69]. Including the Economic Complexity Ratio (lnECR) and Workforce Readiness Ratio (lnWRR) are worth noting as they introduce the concepts of economic complexity and human capital into the equation. These variables also demonstrate intricate connections with financial metrics, indicating nuanced policy interventions are necessary. The incorporation of a wide range of variables contributes to its multifaceted nature [70]. These variables span from Corporate Environmentalism to Economic Complexity and Workforce Readiness [71]. It further supports the idea that evaluating sustainable supply chains is a complex process influenced by various factors, including economic, environmental, and social aspects [72]. In summary, your research serves as an essential foundation for future inquiries into the intricate dynamics of these variables, particularly within the unique context of sports stadiums [73]. It also lays the groundwork for future policy development and research.

## 5. Conclusion and policy implications

### 5.1. Conclusion

This study provides a comprehensive analysis of sustainable supply chain management within sports stadium ecosystems, focusing on the Shanghai region in China and using data from 2008 to 2022. By employing the Method of Moments Quantile Regression (MMQR) model, the research uncovers the intricate relationships between Corporate Environmentalism (CE), Population Density (PD), Economic Complexity Ratio (lnECR), Workforce Readiness Ratio (lnWRR), and Gross Domestic Product (GDP) differentiation. The findings emphasize the unique challenges of achieving sustainability in sports stadiums, which are characterized by their high resource consumption and economic activity. The study demonstrates the significance of geographical and demographic factors in influencing these relationships, as demonstrated by the significance of Population Density. In addition, it highlights the intricate and interdependent relationships between Corporate Environmentalism and economic indicators, adding a level of intricacy to policy discussions surrounding sustainable development. The study’s findings are particularly significant in sustainable supply chain valuation, specifically in the context of sports stadiums. This sector, although niche, has a significant social and economic impact. The study provides valuable insights into the connections between the variables being evaluated. Also, it highlights the need for additional research to explore these connections’ intricate and conditional nature. The findings call for reevaluating policy approaches to achieve sustainable development, promoting a more nuanced and multi-dimensional strategy. This research provides valuable insights for stakeholders in sports stadiums and beyond, offering practical guidance on balancing economic growth with environmental sustainability. It goes beyond being just an academic exercise and offers actionable recommendations. The study uncovers a complex connection between Corporate Environmentalism (CE) and Gross Domestic Product (GDP) differentiation. The evidence to support an association between corporate environmentalism and economic outcomes, the data indicates that higher levels of environmentalism in businesses could potentially lead to less variation in GDP. This discovery is groundbreaking as it prompts us to reconsider the conventional story surrounding the clash between preserving the environment and fostering economic development.

### 5.2. Policy recommendation

The complex relationship between sustainable supply chains, environmental outcomes, and the varied economic impacts in sports stadiums has revealed numerous significant findings. First and foremost, it is clear that sports stadiums, as important cultural hubs, significantly impact the economy and the environment. The study findings highlight the importance of implementing flexible and tailored policy interventions due to the complex relationships and non-linear patterns observed in the variables. The results emphasize the significance of encouraging sustainable practices within stadiums. Considering the notable impact of population density (PD) on GDP differentiation, it is crucial to consider urban planning around sports venues carefully. Policymakers should consider the population dynamics, particularly in densely populated areas, and prioritize the development of efficient transportation and infrastructure to mitigate potential environmental challenges. The study suggests that as we navigate the intricacies of economic indicators such as the Economic Complexity Ratio (lnECR) and the Workforce Readiness Ratio (lnWRR), there is a strong need to enhance educational and skill development programs. Considering the complex economic situation, efforts like these, designed for stadium management and its stakeholders, would create a significant setting for sustainable supply chain management. The conditional relationships, especially the interaction between Corporate Environmentalism and GDP differentiation, suggest a requirement for policy incentives based on specific conditions. A well-rounded strategy that considers economic and environmental factors could be achieved by implementing policies that offer increased advantages to stadiums that strike a commendable balance. Policymakers need to consider the clear trade-offs, particularly regarding different levels of GDP differentiation. The importance of stakeholder collaboration cannot be emphasized enough.

### 5.3. Limitations and future research directions

Despite its significant contributions, this study has several limitations that offer avenues for future research. First, while the analysis focuses on the Shanghai region and uses data spanning from 2008 to 2022, the findings may not be directly generalizable to other regions with different economic, demographic, and environmental characteristics. Future studies could expand the geographical scope to include diverse regions, particularly developing economies, where sports stadiums may face unique challenges in implementing sustainable supply chains. Second, the reliance on historical data assumes a degree of stability in economic and environmental variables, potentially overlooking the dynamic and rapidly evolving nature of supply chain ecosystems influenced by technological advancements, policy changes, and global disruptions such as pandemics or climate-related events. Incorporating real-time or predictive data analytics into the framework could enhance the adaptability of the proposed model.

Additionally, while the study employs the Method of Moments Quantile Regression (MMQR) to capture conditional and non-linear relationships, the model assumes a static relationship between the variables over the study period. Future research could explore dynamic modeling approaches, such as time-series or panel data analysis, to account for temporal variations and interactions. The study also primarily focuses on macroeconomic and demographic factors, leaving out other critical dimensions such as technological readiness, consumer behavior, and regulatory frameworks, which could significantly impact the adoption and effectiveness of sustainable practices. Future work could integrate these dimensions to provide a more holistic understanding of sustainability in sports stadium ecosystems.

Finally, this study highlights the trade-offs between economic and environmental objectives, particularly at higher GDP differentiation quantiles, but does not delve deeply into strategies to mitigate these conflicts. Future research could investigate specific policy interventions, such as incentives for green technologies or community engagement programs, to balance these objectives more effectively. Moreover, exploring the sustainability dynamics across different types of sports facilities, events, and operational scales could provide further insights into tailoring strategies for diverse contexts. These directions would not only build on the findings of this study but also contribute to the broader discourse on sustainable supply chain management in complex and high-impact sectors.
